# The Analysis of the Effect of Blood Transfusion on Changes of Blood Platelet Parameters in Patients with Leukemia Treated with Chemotherapy

This article has been retracted.

**DOI:** 10.1155/2022/2901993

**Published:** 2022-08-29

**Authors:** Yangxin He, Shanshan Liang, Yali Xu, Chunjing Wan, Feng Ma, Baoyan Wang

**Affiliations:** Department of Blood Transfusion, The First Affiliated Hospital of Xi'an Jiaotong University, Xi'an 710061, Shannxi, China

## Abstract

**Objective:**

To study and analyze the effect of blood transfusion on the change of blood platelet parameters in patients with leukemia treated with chemotherapy.

**Methods:**

Ninety-eight patients with leukemia treated with chemotherapy in the First Affiliated Hospital of Xi'an Jiaotong University from January 2021 to January 2022 were selected to observe the changes of platelet parameters before and after blood transfusion.

**Results:**

There was significant difference between pre-transfusion and post-transfusion indexes (platelet count, mean platelet volume, and hematocrit) (*P* < 0.05). After binary logistic regression analysis, the use of antibiotics (OR = 2.235), blood transfusion history (OR = 3.086), abnormal white blood cell count (OR = 1.134), and frozen plasma transfusion (OR = 3.121) were the main factors of blood platelet parameters after transfusion in leukemia patients (*P* < 0.05).

**Conclusion:**

Blood transfusion is beneficial to improve blood platelet parameters and prevent bleeding in patients with leukemia treated with chemotherapy. Attention should be paid to patients with risk factors for poor response to blood platelet transfusion and early intervention.

## 1. Introduction

Acute leukemia is a malignant clonal disease of hematopoietic stem cells. Abnormal proliferation of primitive and immature cells inhibits normal hematopoiesis of bone marrow and can also infiltrate extramedullary organs such as the liver, spleen, and lymph nodes. It is mainly divided into two types: acute lymphoblastic leukemia and acute myeloid leukemia [1], and the mortality is high in malignancies [2]. To prevent thrombocytopenia or bleeding, blood transfusion therapy is one of the supportive care measures for leukemia patients following cytotoxic chemotherapy [3, 4]. However, during blood transfusion therapy, the body is stimulated to produce anti-platelet-associated antibodies due to the immune effect of leukocytes in blood products, affecting the effect of platelet transfusion, resulting in no significant increase in platelet count, bleeding symptoms are not significantly controlled, fever, allergy, and other adverse reactions may also occur, and intracranial hemorrhage may also be caused in severe cases [5, 6]. At present, there is no unified theory about the changes of platelet coefficient and related influencing factors after blood transfusion treatment, and there are few related studies. Therefore, it is of great significance to identify the effect of blood transfusion on blood platelet parameters in leukemia patients treated with chemotherapy as early as possible and take effective intervention in a timely manner.

## 2. Study Subjects and Methods

A total of 98 leukemia patients who were treated with chemotherapy in the department of hematology from January 2021 to January 2022 in the First Affiliated Hospital of Xi'an Jiaotong University were selected by convenience sampling. All patients were diagnosed by bone marrow examination and met the Criteria for the Diagnosis and Efficacy of Hematological Diseases. Chemotherapy regimen is in line with the National Comprehensive Cancer Network (NCCN) guidelines for adult leukemia treatment. All patients received adjuvant treatment with traditional Chinese medicine. Compound ingredients: Angelica sinensis, Astragalus membranaceus, Ligustrum lucidum, Atractylodes macrocephala, Radix Pseudostellariae, Radix Scutellariae, Radix Polygoni Multiflori, wolfberry, dodder seed, Fructus Psoraleae, Morinda officinalis. The patient took the prescription orally once in the morning and once in the evening. This study was approved by the medical ethics committee of the First Affiliated Hospital of Xi'an Jiaotong University (no. xjt122), which is in line with the Declaration of Helsinki. All patients signed informed consent.

### 2.1. Inclusion Criteria

Inclusion criteria were as follows: (1) patients who signed the informed consent form of blood transfusion products and (2) patients having clear consciousness.

### 2.2. Exclusion Criteria

Exclusion criteria were as follows: (1) combined with other diseases that can lead to thrombocytopenia such as malignant tumors, rheumatism, and immune system diseases; (2) combined with important organ dysfunction; (3) patients with mental disorders who cannot cooperate with this study; and (4) breastfeeding or pregnant women.

### 2.3. Methods of Blood Transfusion

Whole blood and blood components were all included. According to the specific implementation of conventional chemotherapy regimen, when the patient developed clinical abnormalities after chemotherapy, multiple transfusions of whole blood were required, each transfusion volume was 300 ml, blood was transfused every other day for 3 consecutive transfusions, and another 10 U therapeutic dose of blood platelets was transfused.

### 2.4. Outcome Measures

Baseline data such as gender, age, disease type, antibiotic use, history of blood transfusion, and platelet type (frozen platelets and fresh platelets) were collected. Within 24 hours after the end of chemotherapy, 2 ml of fasting peripheral venous blood was extracted with EDTA anticoagulation tube. Platelet count (PLT), mean platelet volume (MPV), platelet volume distribution width (PDW), and platelet volume (PCT) were measured by automatic blood cell analyzer within 24 hours. The corrected count of increment (CCI) was calculated. CCI = (post-transfusion platelet count transfusion-pre-platelet count) (10^9^/L) × body surface area (m^2^))/(total number of platelets transfused (10^11^/L)). If the CCI value at 24 hours after transfusion was less than 4.5 × 10^9^/L, it indicated that the platelet transfusion was ineffective.

### 2.5. Data Analysis

Data analysis was performed using the software SPSS 24.0, expressed as mean ± standard deviation, qualitative data were described as percentages, and quantitative data were tested by normality. The platelet correlation coefficient of patients before and after blood transfusion was compared by paired sample *t*-test. Binary logistic regression analysis was used to analyze the influencing factors of platelet transfusion efficacy. *P* < 0.05 indicated a statistically significant difference.

## 3. Results

### 3.1. Baseline Characteristics

This study included 52 cases of acute lymphoblastic leukemia (ALL), 22 cases of acute myeloid leukemia (AML), and 24 cases of acute promyelocytic leukemia (APL). The mean age of patients was 42.13 ± 1.02 years old (range 34 to 69 years old), males accounted for 44.9% (44/98), antibiotics were used in 38.8% (38/98), frozen plasma was transfused in 20.4% (20/98), and white blood cell count was abnormal in 24.5% (24/98). Patients who had a blood transfusion history before this transfusion accounted for 42.9%, 32 patients developed clinically abnormal changes during the chemotherapy period, and 66 patients developed clinically abnormal changes during the interval between chemotherapies (within 2 weeks after the end of the chemotherapy course), and 15 patients did not respond to platelet transfusion.

### 3.2. Changes in Blood Platelet Parameters before and after Transfusion

Comparative analysis of blood platelet parameters before and after transfusion showed that MPV, PCT, and PLT were significantly improved in patients after transfusion, as shown in Table 1.

### 3.3. Influencing Factors of Blood Platelet Parameter Changes after Transfusion

The CCI value at 24 hours after transfusion was bounded by 4.5 × 10^9^/L to determine whether this blood platelet transfusion was effective or ineffective, and the CCI value at 24 hours was used as the outcome measure. Among all the patients, 15 patients who failed to respond to transfusion were selected, and 15 patients were randomly selected in a ratio of 1 : 1 among 83 patients who responded to transfusion for secondary analysis. Binary logistic regression analysis showed that the use of antibiotics, history of blood transfusion, abnormal white blood cell count, and frozen plasma transfusion were the main factors affecting the changes of blood platelet parameters after transfusion in leukemia patients (*P* < 0.05), as shown in Table 2.

## 4. Discussion

Leukemia is a clonal malignant disease with abnormal hematopoietic stem cells, which has a great impact on the life safety of patients. Clinical manifestations of patients were anemia, infection, severe bleeding symptoms, and death in severe cases. At present, chemotherapy is mainly used to improve the clinical symptoms of patients in clinical practice, mainly to change blood platelet parameters, and specific treatment is carried out [7]. Different degrees of bleeding caused by thrombocytopenia in patients with leukemia after chemotherapy are the main factors leading to death. Blood transfusion is currently one of the common methods to treat and prevent bleeding in patients with acute leukemia. However, in repeated blood transfusion, bone marrow megakaryocytes divide and proliferate, significantly reducing the effect of blood transfusion [8]. Adverse reactions of blood transfusion may occur, which can seriously interfere the therapeutic effect and lead to various serious consequences such as blood transfusion lung injury and pulmonary microvascular embolism, increasing the risk of death [9]. Exploring the changes of blood platelet parameters and influencing factors in patients with leukemia treated with after blood transfusion and giving targeted suggestions are the key to guide the planning of treatment options and improve the therapeutic effect.

In this study, patients with leukemia treated with chemotherapy received blood transfusion treatment, including whole blood transfusion and blood components. The main purpose was to prevent bleeding and regulate platelet-related parameters. MPV, PCT, and PLT were significantly different before and after transfusion, which indicated that blood transfusion could improve blood platelet parameters and prevent bleeding in patients with leukemia received chemotherapy. This finding is partially in contrast to the findings of Comont et al.'s study [10], which showed that in multiple transfusions, patients developed platelet antibodies, PCT and PLT gradually decreased, and MPV gradually increased. Although transfusion of whole blood and component blood can bring obvious therapeutic effect, it affects the therapeutic effect due to the complex components of blood products [11].

At present, the effect of blood transfusion on blood platelet parameters in patients with leukemia who received chemotherapy is influenced by multiple factors, but the results of various studies are not uniform [12, 13]. In this study, the results of binary logistic regression analysis showed that the use of antibiotics, history of blood transfusion, abnormal white blood cell count, and frozen plasma transfusion were the main influencing factors of ineffective platelet transfusion after blood transfusion in leukemia patients. However, there was no significant difference regardless of age or gender. Leukemia patients can be affected by a variety of factors, causing fever, infection, and other complications, requiring the use of antibiotics, resulting in a large number of platelet consumption. Inflammatory reactions can produce a variety of antibodies, resulting in rapid reduction of platelet counts and affecting platelet transfusion [14]. Frozen blood platelets increase the risk of exposure to phosphatidylserine moieties during freezing, prompting platelet activation, which in turn accelerates the rate at which blood platelets damage the mononuclear phagocytic system after entering the body, resulting in insignificant improvement in blood platelet counts and poor response to transfusions after treatment with blood platelet transfusions [15]. The study by Tantanate et al. [16] indicated that multiple blood platelet transfusions resulted in decreased platelet counts and increased risk of bleeding, similar to the finding that a blood transfusions history was a risk factor for platelet transfusion efficacy in this study. Research [17] showed that when patients receive platelet infusion, leukocytes in the body can secrete a large number of histamines, leukotrienes, and other components, which promote the body to have allergic reactions, increase the risk of hemolysis and allergy, and then affect the effect of infusion treatment, which is similar to the result that abnormal leukocytes increase the risk of ineffective infusion in this study. The sample size of this study is less, which may affect the authenticity of the results. The research is still limited, and large-sample research is needed to explore and analyze.

## 5. Conclusion

Blood transfusion is beneficial to improve blood platelet parameters and prevent bleeding in patients with leukemia treated with chemotherapy.

## Figures and Tables

**Table 1:** Changes in blood platelet parameters before and after transfusion.

	MPV (fL)	PDW (%)	PCT (%)	PLT (×10^9^/L)
Pre-infusion	10.39 ± 0.68	16.17 ± 0.03	0.024 ± 0.005	55.90 ± 0.16
24 hours after infusion	10.23 ± 0.79	16.23 ± 0.05	0.053 ± 0.004	60.08 ± 0.92
*T*	−5.397	−2.359	−15.158	−9.469
*P*	0.006	0.078	<0.001	0.001

**Table 2:** Influencing factors of blood platelet parameter changes after transfusion.

	*B* value	Standard error	Wald value	OR	95% CI	*P* value
Gender	0.731	0.671	2.537	4.105	2.147–8.092	0.347
Age	0.257	0.833	17.246	7.136	4.099–10.765	0.134
Antibiotic use	0.804	0.645	1.552	2.235	0.631–7.918	0.213
History of transfusion	2.674	0.746	11.412	3.086	2.766–5.908	0.007
Abnormal white blood cell count	3.705	0.842	19.673	1.134	0.91–2.419	0.001
Platelet species	1.788	0.564	10.335	3.121	2.034–8.132	0.03

## Data Availability

The data used to support the findings of this study are available from the corresponding author upon request.
